The article "Dilemma and Solution of Copyright Justice System for Health Short Video under Network Big Data Environment Monitoring" was retracted in 2023. Reasons: unreliable results or conclusions; concerns about the data; concerns about the peer review; concerns about the citations.

# Dilemma and Solution of Copyright Justice System for Health Short Video under Network Big Data Environment Monitoring

**DOI:** 10.1155/2022/9640574

**Published:** 2022-10-05

**Authors:** Fangfang Li

**Affiliations:** Pingdingshan University, Pingdingshan 467000, China

## Abstract

Short videos have quickly taken over the mobile screens of network users and established themselves as one of the most significant social platforms in the “Internet+era” as a new carrier of social culture. Short films have the qualities of high participation, strong engagement, high real-time, and quick propagation, which satisfy the needs of Internet users in interpersonal communication and reading or enjoyment in leisure time. This is against the backdrop of network big data environment monitoring. Based on this, the paper defines the fair use system of short video copyright, elaborates on its concept, examines the system's challenges and potential fixes in the context of networks, and develops a model for short video repeat detection using local key points. According to the experimental findings, this algorithm's short video repetition detection accuracy rate can reach 95.8%, and its recall rate can reach 94.5%. For the development of the fair use system of short video copyright in the current network environment, the video in some complex scenes can achieve good detection performance, which establishes a good data analysis foundation and provides a significant amount of assistance for the system to escape its predicament.

## 1. Introduction

From popular blogs to podcasts, from PC video websites to the new generation of short video social platforms, the evolution of mainstream entertainment has witnessed the changes in the expression of Internet content. Thanks to the development of mobile communication technology and the popularity of portable terminal equipment, short video, as a new carrier of social culture, has formed a blowout development in a short period of time, rapidly seizing the mobile screen of network users, and has become one of the most important social platforms in the “Internet+era” [1]. During the Spring Festival epidemic in 2020, the playing type of short videos was favored by users, accounting for 68.4% [2]. In the last two years, the development of short videos has become stronger, and it has become the best choice for leisure and entertainment and an important channel for people to obtain network information [3]. The reason why short videos develop so vigorously is driven by many factors. In terms of policy, the relevant departments of the state have made great efforts to rectify. In terms of development, all major platforms actively expand overseas. In science and technology, the Internet technology is constantly innovating and developing. In terms of content, big data brings viewers a more high-quality and refined impression [4]. Nowadays, short videos are becoming more and more diversified. The long-term development of “short videos” has great commercial value and development potential. The short video market has considerable prospects in the future. The sprouting of short video social platform originated from Viddy, a software in the United States, which allows its users to directly upload videos created by themselves to social platforms by connecting with major mainstream social platforms such as Twitter and Facebook. At the same time, major short video social applications in China have sprung up like bamboo shoots, and apps such as Kwai, Tiktok, and Meipai have stood out in the fierce fight [5, 6]. In 2017, short video content creators represented by Papi sauce sprang up, and the short video industry ushered in the spring. Short video users in China have reached approximately 600 million, or 42% of the country's total population and 74.1% of all Internet users, according to the 2018 Research Report on China's Online Visual Tracking Development [7]. However, behind the prosperity and growth of short videos, due to the imperfect copyright protection, they have fallen into the mire of piracy and infringement. Disputes about the copyright of short videos emerge one after another. Whether short videos can enjoy the copyright is not only a gap to be filled in theory, but also a focus of debate in judicial practice.

Short films have the qualities of high participation, robust engagement, high real-time, and quick propagation against the backdrop of Internet big data, which meets the needs of Internet users in interpersonal communication and reading or amusement in leisure time. By granting them the sole authority to regulate the dissemination of works, copyright laws safeguard the legal interests of copyright holders in the conventional setting. However, this power is not a total monopoly and needs to be constrained to a certain extent. The copyright law establishes a fair use system to maintain the equilibrium between the personal interests of copyright owners and the interests of the social public [8]. It cannot obstruct either the normal dissemination of works or the normal contact of the social public with works. This interest balancing pattern has been broken in the network environment. On the one hand, a lot of works have been uploaded to the Internet for free distribution and use, violating the copyright owner's exclusive control over the works, thanks to the ease of network communication and the low cost of copying. The copyright owner has reported the network infringement in order to defend their own interests, but has run against the defence of legitimate use [9]. On the other hand, copyright owners use private remedies to protect their rights, primarily through the use of technical controls to restrict access to and dissemination of works. This prevents authorised users from accessing the works without having a reasonable opportunity to use them and denies them information. This severely restricts the distribution and efficient use of social and cultural resources, as well as denying the public the right to regular access to works [10]. Facing the challenge of the network environment, the traditional system has encountered the dilemma of choice, and it is urgent to adjust the current system to find a correct way to keep up with the development of the network era [11]. Studying the conundrum and solution of the reasonable use system of short video copyright under the network big data environment is therefore of far-reaching significance for safeguarding the legitimate rights and interests of copyright owners and fostering the healthy and sustainable development of the cultural industry.

The short video repetition detection algorithm based on local key points in the network big data environment is examined in this research, along with the challenges and solutions of the fair use system of short video copyright. Beginning with the definition and attributes. The video similarity measuring method's algorithm has been improved, and it now has good detection performance for videos with complicated scenes. For the creation of a short video copyright fair use system in the current network environment, it creates a solid data analytic base. In order to maintain the copyright of short videos, it can also offer a strong confirmation of detection findings.

A short video repeat detection model based on local key points is created and examined by evaluating the backdrop of the conundrum and the solution of the fair use system of short video copyright in the network big data environment. The primary contributions and innovations of this paper are:

1. For the innovation of the topic selection, by combining the difficulties and solutions of the network big data environment and the fair use system of short video copyright, the traditional fair use system of copyright has been enriched. Based on this background, it is an innovation to explore the difficulties and solutions of the fair use system of short video copyright. This paper also analyzes the model and hopes that the discussion can help the fair use system of short video copyright out of the dilemma
2. In this paper, we use the shot level comparison and the network video repetition detection method for reference. Firstly, a new global feature shot signature is defined at the shot level, and on this basis, a video repetition detection method based on accurate nearest neighbor search based on shot level comparison is proposed. This method can judge the similarity of videos by the ratio of matched shots between videos
3. In this paper, in order to further improve the speed of finding similar shots, on the basis of the video repetition detection method of accurate nearest neighbor search based on the comparison of local key points in the shot layer, the famous approximate nearest neighbor search technology is used to quickly find similar shots in the shot layer, and a short video repetition detection method based on local key points is proposed

## 2. Related Work

With the quick advancement of digital technology, many academics have joined the debate over copyright protection for short videos. Lee M J et al. discussed the originality of short videos, the recognition of reasonable use and the legal liability of the communication platform, especially made a detailed statement on the original short videos, and believed that the copyright legal rules applicable to general film and television works could not be directly applied to the issues related to short videos [12]. When Vizireanu P D N analyzed the path between the originality of short videos and the protection of copyright law, they believed that although the selection space of short videos was small and the time was short, they might still be original and obtain the protection of copyright in a narrow sense as audio-visual works. Based on the narrow sense of copyright and performer's rights, the right holders of short videos can be fully protected under the framework of the current law without any modification to the system [13]. The definition of this concept mainly highlights the functional attribute of reasonable use, i.e. “use,” which is the use without consent and without compensation. Jiang Jie et al. proposed that “reasonable use refers to the use of copyrighted works without the consent of the obligee, generally without payment, and does not constitute infringement.” However, the word “general” is slightly general and does not express the premise that reasonable use requires legitimate reasons [14]. Wakata S et al. reasonable use is “a legal act of using other people's copyright works for legitimate purposes without the consent of the copyright owner and without paying compensation to the copyright owner under the conditions prescribed by law.” This concept comprehensively describes the connotation and extension of fair use, and emphasizes that the act of fair use should be a legal factual act from the perspective of behavior characterization. However, this concept also has some disputes on the selection of objects. The object of reasonable use is regarded as the work itself, and the object of reasonable use should be the right of the copyright owner [15]. Spelten E R et al. believe that in the collective information management system of copyright information, in addition to the personal information of the obligee, the monitoring system attached to the management system will also involve the private domain of the user to some extent [16]. Through the research on the fair use of short video works, Chan H Y et al. He believed that it brought new challenges to the fair use system, such as the expansion of copyright, the reduction of the scope of reasonable application, and the difficulty in distinguishing fair use from infringement and piracy [17]. Zhang Wenwei et al. proposed that the ID watermark of the short video user can be recognized as the specific performance of the short video creator's signature right. Although the watermark of the short video platform can not indicate the ownership status of copyright and can not be recognized as the exercise of the right of authorship, it shows the identity of the disseminator of the short video platform in the process of work dissemination and can be recognized as the right management information [18].

The virtual, paperless, and information-based characteristics of the network itself have created the complexity and diversity of the new challenges faced by the conventional copyright fair use system, despite the fact that some scholars have begun to investigate this aspect due to the network's rapid development. In addition, the study is not thorough, in-depth, and specialised, and the regulation is rigid, which makes it impossible for the fair use system to adapt to the advancement of contemporary science and technology. Currently, there are also few researchers interested. Scholars from both home and abroad are currently less involved in the development and operation of the network environment's fair usage system. As a result, the judge's discretion in actual court proceedings is constrained, copyright dispute cases are nonexistent, and there is no money available for their pursuit. Given this, the author thinks it is imperative to talk about the problem and solution of the short video copyright fair use system in the network context. This system is a significant development that affects the fundamental rights of copyright holders, users, and distributors as well as the state of intellectual property law and research. This paper explains the idea of fair use of copyright and defines and describes short videos based on the pertinent definition of this system. It examines the system's problems and potential solutions in the context of the network environment and builds a short video repeat detection model based on regional important points that significantly aids the system in overcoming its challenges.

## 3. Methodology

### 3.1. Definition of Fair Use System of Short Video Copyright

#### 3.1.1. The Concept of Fair Use of Copyright

The common law nations are mostly those that use the fair use approach of copyright. The word “copyright limitation” is not typically used in civil law countries' legislation; instead, the system is described as such. In academic communities across the globe, the fair use system of copyright has always been a perplexing and contentious subject [19]. This emphasis accurately captures the overall balance of copyright laws everywhere. The perpetual conundrum of copyright law determines the end of the owner's exclusive right and the beginning of the public's access to freedom of works. Any system could be seen of as having been created to address the issue of interest balance [20]. The fair use system is required by law in order to strike a balance between copyright owners' rights and societal concerns. It is possible to see the legal foundation of this system as a limitation on the freedom enjoyed by copyright holders. The law requires the copyright owner to fulfil certain obligations for society in addition to protecting the legitimate rights and interests of the copyright owner. This prevents the copyright owner from having an absolute monopoly over the rights, advancing the progress, and development of the entire society.

#### 3.1.2. Definition, Characteristics, and Classification of Short Video

As for the definition of short video, there is no clear definition in the academic circles. At present, the definition of short video mainly includes the following: (1) short video refers to a new type of real-time video sharing form that is recorded, edited, and uploaded on some special short video platforms with seconds as the counting unit, and the audience plays on this platform. (2) Short video is different from long video; in that, it is played on new media, which is more convenient for dissemination and sharing, and the duration is usually within five minutes. (3) Short video refers to a new video format in which the video content is shorter than 15 minutes, which is more spread and photographed by Internet mobile intelligent terminals, beautified and edited by Internet mobile intelligent terminals, and the video is shared to social media platforms in real time [21]. Other mainstream media also define short video as “video content transmitted by PC and mobile devices with playing time less than 5 minutes”. To sum up, short video refers to a new video form completely different from traditional long video, which is limited in length and automatically recorded, edited and created by users of social platforms, and then uploaded to social platforms to realize information sharing, communication, and dissemination.

Compared with the traditional long video, the short video is characterized by the following three points: first, the propagation speed is fast and the range is wide. The traditional long video transmission has a natural lag. However, the duration of the short video is usually controlled from a few seconds to a few minutes. In today's fast-paced and fragmented lifestyle, short videos break through the limitations of time, space, and people, acquire information in a more intuitive and convenient way, conform to the browsing trend of modern people, make full use of the fragmented time, and accelerate the dissemination of information. Second, the production threshold of short videos is low and the review process is simple. The production cycle of traditional long videos has become longer, and the production cost is high. In the process of uploading and publishing after the production is completed, the review of its content and quality is also relatively strict. The time to make a short video is short, and a mobile phone can complete the entire production process, and can shoot and share at any time, greatly reducing the threshold of video production. At the same time, the self-contained beauty, filter, special effects, and other functions of the short video application also make it easier and faster for users to express their personal ideas freely. Third, short video information points are prominent and in line with the current trend. The traditional long video does not refine the story enough. Due to the short time length and limited creative space, the short video makes the information content more focused and distinct, which can make the audience quickly understand the theme and easily resonate. For the current events, they can be conveyed in the form of short videos in a timely manner, which is conducive to the dissemination of current thoughts and emotions, and promotes the diversity of cultural communication.

At present, there are many kinds of short videos, and there are many platforms. There are three common categories: first, according to the characteristics of content producers, short videos can be divided into UGC, PGC, and PUGC by using Internet terms. As shown in Figure 1, this classification method can be understood more vividly.

UGC is “user original content” or “user produced content”. The short video under this mode has a large number of users, high upload freedom, and strong flow adsorption, but the video content quality is uneven, the user viscosity is low, and the realization mode is unclear. Such platforms as Youtube, Tiktok, and Kwai are mostly producers of such content. PGC is “professional production video short video”, which refers to the video carefully produced by professionals with professional shooting knowledge and working experience. Compared with the UGC Internet short videos, the short video content created by them is of higher quality and professional. For example, Wanhe Tianyi, which is famous for its “wanwan unexpected series”, and Li Ziqi, whose team is characterized by displaying rural scenery, have formed their own brand effect, which can lay a foundation for subsequent drainage and realization, and thus become an important choice for seeking new business development in the “Internet+era”. A content production mode combining PGC and UGC is known as PUGC, or “professional users produce content.” The brief movie in this mode combines the two benefits of PGC and UGC, and it adopts the universality of PGC and professionalism of UGC as a defining technique to draw in and compel users. Examples of platforms that primarily produce this kind of material include dragonfly FM, watermelon video, good-looking video, and others.

Second, according to the functional characteristics of the content, short videos can be divided into social, information, and tools. The social category is represented by “Tiktok”, “Kwai”, “Weishi”, and “Wechat video Number”. This type of short video has a large number of users, strong stickiness, and wide utilization rate. In addition to the main shooting functions, it also has the functions of attention, praise, making friends, and private messages, and has typical social attributes. Third, according to the characteristics of content originality, short videos can be divided into original and secondary creation. Most of the original videos are short videos created with practical skills, street interviews, short sitcoms, etc. in the selection and expression of materials, music, scenes, and subtitles, these short videos reflect the “personalized expression” of the producer, which brings different feelings to the audience and can be distinguished from other short videos. For example, the short video “Siping police incident” series stories. The secondary creation category is mainly short videos created with film review introduction, game interpretation, creative imitation, etc. such short videos are created on the basis of the existing works of others, such as the short video “Gu amo” series film review, by means of serial burning, mixing, and cutting, parody, etc.

### 3.2. Analysis on the Dilemma and Solution of the Fair Use System of Short Video Copyright under the Network Big Data Environment

After the emergence of digital network technology, this situation has gradually changed. The large-scale unauthorized use of works on the Internet has greatly affected the interests of obligees, and to a certain extent led to the shrinkage of traditional video, books, and other industries. Therefore, both the copyright owner and the copyright industry must examine the traditional thinking mode. The traditional “closed” protection mode aiming at reducing illegal use should be changed to the “open” protection mode aiming at increasing legal use. Facing the massive short video works on the Internet, copyright owners and users need an efficient and low-cost way to authorize the use of works, which requires finding a way to market the large-scale use of short video works on the Internet. China's regulations on the protection of the right to information network dissemination states in paragraph 1 that “in order to protect the right to information network dissemination, the obligee may take technical measures,” while paragraph 2 states that “no organisation or individual shall intentionally avoid or destroy the technical measures, and shall not intentionally manufacture, import, or provide the public with devices or components that are mainly.” In actuality, copyright owners frequently abuse and overuse network technological measures, which significantly lowers the scope of reasonable use of copyright and prevents the public from sharing public knowledge.

The fair use system's value objective is to advance scientific and cultural endeavours by balancing the rights of copyright holders, communicators, and the general public. Therefore, this approach has been formed in all nations' copyright laws or legal procedures.

The legal principle is the core content and guiding element of the legal structure. It is the sustenance of the spirit and soul of the legal structure. It makes the legal institution itself more reasonable and perfect and more adaptable, and guides the creation and specific application of the legal rules. The social values and social situation will change under certain conditions, and the legal principles will be adjusted and changed accordingly. Therefore, in order to deal with various problems brought by entering the era of digital copyright, China's fair use system rules should follow the following basic principles when revising: first, the principle of balance of interests. Second, we should combine our national conditions, learn from foreign advanced technologies, and conform to the trend and principles of international copyright legislation. Third, appropriately expand the scope of reasonable use and improve the standards and principles for the identification of infringement of online works. In the specific process of improving the fair use system, China should take the above principles as the basis and guidance. These principles complement each other, are inseparable, and are indispensable. Only by correctly grasping these principles can we ensure that the rules formulated conform to the legitimacy and rationality, thereby injecting new blood into the traditional fair use system and withstanding the challenge of digital technology.

### 3.3. Construction of Short Video Repeat Detection Model Based on Local Key Points

For the duplicate detection model of short video, the user refers to a query seed video, and automatically queries the video database for similar or duplicate videos with the content of the seed video. The video data processing layer mainly includes three components: shot boundary detection, feature value extraction, and feature value matching. These three components provide corresponding interface calls for the server to complete the core work of the short video repetition detection algorithm. The video data processing layer in this system is written in language, and the technology used to complete the interaction between the server and the short video data processing layer. The data persistence layer mainly includes two databases: short video file database and system database. We know that the data volume of general video files is relatively large. If it is saved in the database, it will inevitably consume a lot of time and affect the efficiency during video reading. Therefore, this system uses the file system to save the video data. We only need to record other description information of the video file and the storage address of the video file into the system database. The overall framework of the detection system is shown in Figure 2.

A practical application of the network video repetition detection algorithm is also an exploration of the development direction of the video sharing website. The project scope is small, and the database design of the system is not large and complex. Therefore, we choose MySQL database management system with small volume, high speed, and low cost as the database of the system. MySQL is a small relational database management system. The system includes four tables in total: user table, video information table, user video relationship table, and video shot feature table. We use the graph entity relationship diagram to describe the attributes of the table and the relationship between the tables, as shown in Figure 3.

The general video is composed of multiple shots through splicing and editing. Shot is the smallest semantic unit of video data. It is a continuous frame sequence in time or space captured by a camera, representing a group of continuous actions. Shot is the basic unit of video and the basis for in-depth analysis of video. Shot boundary detection is actually to divide the video file into independent shots. We use *H*_*k*_ = (*h*_*k*1_, *h*_*k*2_, ⋯*h*_*kd*_) to represent the color histogram of the second frame of the video. The distance between two adjacent frames is defined as:

(1) $$\begin{array}{c} D\left(H_{k},H_{k+1}\right)=\sqrt{\overset{d}{\underset{i=0}{\sum }}{\left(h_{k1}-h_{\left(k+1\right)}i\right)}^{2}}. \end{array}$$

The shot boundary detection algorithm based on color histogram is to use the characteristics between shots to project the value of each point of the video frame into a small discrete interval, then count the number of pixel points in each cell in the interval, and use the distance between two adjacent frames using European distance technology. If the distance is greater than the set threshold, the frame is considered to be at the shot boundary, and the sequence number of the video frame is returned as the starting position of the shot. Otherwise, the calculation continues. The distances between lens features are as follows:

(2) $$\begin{array}{c} Dis\left({SS}_{i},{SS}_{j}\right)=\sqrt{\overset{d}{\underset{k=1}{\sum }}{\left({SS}_{ik}-{SS}_{jk}\right)}^{2}}, \end{array}$$

where represents the feature value of the *SS*_*i*_ lens, *d* is the dimension of the lens feature, and *SS*_*jk*_ represents the value of the *k* dimension of the lens feature value. The shot boundary detection method based on color histogram difference uses the statistical value of pixel color, does not consider the position information of pixels, and only focuses on the global distribution. Therefore, it has strong noise resistance and is insensitive to local object motion. The dimension feature vector is:

(3) $$\begin{array}{c} SS=\left(s_{1},s_{2},\cdots s_{d}\right),s_{i}=\frac{1}{N}\overset{N}{\underset{j=1}{\sum }}h_{ij}. \end{array}$$

Once the features of each shot in the video are extracted, we can compare the similarity of the two shots. One of the main contributions of this paper is to determine whether they are duplicate videos by the proportion of all matched shots between two videos. The more matched shots between two videos, the more similar they are. For better analysis, we define the similarity of videos as follows: “error! Reference source not found” means any video in the database. The expression of its logical function is:

(4) $$\begin{array}{c} F\left(S_{\text{ik}}\right)=\left\{\begin{array}{cc} 1 & \text{if}\underset{S_{\text{ft}\in Vd}}{\min}\;d\left(S_{\text{ik}},S_{\text{jt}}\right)\leq T\\ 0 & otherwise \end{array}\right.. \end{array}$$

Our method can calculate the similarity between the query video and each video in the database within the time complexity by using the technology on the entire data set to obtain the approximate repeated shot set of each shot of the query video. We then fuse these returned repeated shot sets in order to further accelerate the detection speed. This is the precise algorithm:

1. Put the shots of all videos in the database together to build a new data set:

(5) $$\begin{array}{c} D_{s}=\left\{V_{1},V_{2},\cdots V_{N}\right\}=\left\{S_{11},S_{12},\cdots S_{1n_{1}},\cdots S_{{Nn}_{N}}\right\}. \end{array}$$

(2) For each given query shot (point) *S*_*qk*_ ∈ *V*_*q*_. And the threshold *T*. By matching an approximate nearest neighbor set (the shot in the entire data set that matches “error! No reference source found”), the shot is:

(6) $$\begin{array}{c} A_{k}=\left\{S_{1},S_{2},\cdots S_{t_{k}}\right\},k=1,\cdots ,m. \end{array}$$

Among them, *A*_*k*_ ⊂ *D*_*s*_, a video sequence with continuity, and the difference of the estimated depth of the corresponding pixel points in the *h*-dimensional coordinate system should be the same as the difference between their real values. For the image sequence that has undergone time consistent super-pixel segmentation, we use the relative time error to measure the time continuity between the two images:

(7) $$\begin{array}{c} RTE\left(p\right)=\frac{\left|\overset{\wedge }{d_{p}}-d_{p\left(-1\right)}-\left(\overset{\wedge }{d_{p}}-d_{p\left(-1\right)}\right)\right|}{d_{p}}. \end{array}$$

The time consistent super-pixel segmentation algorithm generates a corresponding relationship in the time dimension on the super pixels of consecutive posts. If the corresponding super-pixel pairs marked by the time consistent super-pixel segmentation algorithm between consecutive gaps, the energy function can be expressed as:

(8) $$\begin{array}{c} E\left(d,I\right)=\underset{p\in N}{\sum }{\left(d_{p}-z_{p}\left(W\right)\right)}^{2}+\frac{1}{2}\underset{\left(p,q\right)}{\sum }\left(\alpha^{\left(s\right)}S_{pq}^{\left(s\right)}+\alpha^{t}S_{pq}^{t}\right){\left(d_{p}-d_{q}\right)}^{2}. \end{array}$$

We can calculate the similarity between “error! Reference source not found” and any video in the database by the following method:

(9) $$\begin{array}{c} R\left(V_{q},V_{i}\right)=\frac{\sum_{k=1}^{m}T\left(V_{i},A_{k}\right)}{\left|V_{q}\right|}. \end{array}$$

Wherein,

(10) $$\begin{array}{c} T\left(V_{i},A_{k}\right)=\left\{\begin{array}{cc} 1 & \text{if }V_{i}\cap A_{k}\neq \Theta \\ 0 & \text{if }V_{i}\cap A_{k}=\Theta \end{array}\right., \end{array}$$

*V*_*i*_∩*A*_*k*_ ≠ Θ means that there is at least one shot and seed video in the video in the database. If the *S*_*qk*_ distance of shots is not greater than the threshold value, there must be the most similar shot distance from *S*_*qk*_ to “video error! Reference source not found” not greater than the threshold value.

## 4. Result Analysis and Discussion

The network video stream data used in the experiment are all captured by Wireshark 3 capture software in the campus network environment of Nanjing University of posts and telecommunications. The capture time are April 2022 and May 2022, and the capture time period includes morning, afternoon, and evening. This paper mainly collected seven kinds of video service data, including Tiktok short video, Kwai short video, Youku HD video stream, Microvision, Wechat video number, P2P video (Kankan video), and HTTP video download. A total of 840 video streams were obtained. Each video stream is 3-15 minutes long. Each video stream data is stored in the form of five tuples, including packet arrival time, source IP address, destination IP address, use the protocol type, and package size. The details of the short video data set are shown in Table 1, and the data stream storage format is shown in Table 2.

After obtaining the video stream data, we use the net flow Analab data processing platform to extract the video stream features. The data processing platform is written and built by our team, mainly including batch processing tools (. Bat) and gawk scripts based on line processing text data. In addition, the main data analysis tools used in this paper are Weka and MATLAB 2018a. Weka is an open-source software based on Java programming language, which implements a variety of feature selection algorithms and classification algorithms. It is mainly used for data mining and can be used for data preprocessing, regression, etc. it is a very powerful data mining tool. For several typical statistical characteristics of short video streams, the qualitative analysis of seven types of short video streams is carried out in combination with their distribution maps, and the differences of these characteristics in different types of short video streams are expounded. These features include the mean value of the downlink packet size, the information entropy of the downlink packet size. The characteristic distribution diagram of the downlink average packet size of the seven short video types is shown in Figure 4.

Figure 4 describes the distribution of the average downlink packet size of seven different short video types. It can be seen that the average downlink packet size of Tiktok short video, Kwai short video, Microvision, and Wechat video is large. This is because the server of this type of video mainly transmits a large amount of downlink video data to the user to provide the user with a better viewing experience and service quality. Therefore, more network resources are required for the transmission of downlink data, while the data returned from the client, that is, uplink data, is relatively small, and only some data packets containing control information are sent. In addition, with the improvement of short video definition, the average downlink packet size of the video stream also increases. They are interactive videos and pay more attention to real-time and stability. Therefore, the average size of their downlink packets is relatively small, which is basically kept at about 500 bytes, so as to ensure the interactivity and real-time of the video under the limited network resources. Youku HD video stream and HTTP video at the same time because of the interactivity of these two videos, the number of downstream packets is basically the same. Kankan video is a P2P type video, and the transmission of video stream data will be affected by the sharing node. Just because of this, the average downlink packet size of this type of video will fluctuate violently. The information entropy characteristic distribution diagram of the downlink packet size of the short video is shown in Figure 5.

It can be clearly seen in Figure 5 that only this statistical feature is needed to accurately identify and distinguish Tiktok short videos, which fully illustrates the effectiveness and importance of this statistical feature. In addition, it also shows that the distinguishing ability of a single feature is limited, and it is impossible or difficult to distinguish and identify multiple categories through a single feature, which illustrates the necessity of selecting feature subsets and reflects the importance of feature selection algorithms. In order to analyze the accuracy of video repeat detection algorithms, the speed of various video repeat detection methods is compared, and the comparison results are shown in Figure 6.

In Figure 6, we compare the time taken by various methods to complete the query. It can be seen that the query time based on the algorithm in this paper greatly shortens the running time compared with other methods. The comparison of recall of various short video repetition detection methods is shown in Figure 7.

It can be seen from Figure 7 that the recall of various short video repeat detection methods changes, and the recall of the other two methods is lower than that of the method in this paper. The accuracy of the short video repetition detection method based on this algorithm is the highest, which can reach 94.5%. For those videos with complex scenes, global signature is not enough because dissimilar videos may have similar color distributions. Because there are a large number of repeated videos with different time lengths in the database, the time length is not a very effective feature.  Figure 8 shows the comparison results of the accuracy rate of the repeated detection for short videos.

It can be seen from Figure 8 that the accuracy rate of various short video repeat detection methods changes. The accuracy rate of the short video repeat detection method based on the algorithm in this paper is the highest, which can reach 95.8%. The accuracy rate of the method in this paper is significantly better than the method based on global features, match with the current best key-based method (almost the same). From this analysis, under the same recall rate, the higher the precision rate, the better the performance. In addition, through the use of this technology, the time complexity of this method in the worst case when completing the video repeat detection task is among them, and the retrieval speed is tens of thousands of times higher than that of the method, which can realize real-time detection. The experimental results show that the precision rate of short video repeat detection based on this algorithm can and the recall rate can reach 94.5%. It is concluded that the video with complex scenes can achieve good detection performance, and it establishes a good data analysis foundation for the development of the short video copyright fair use system in the current network environment. It can also provide a good proof of detection results for the maintenance of copyright of short videos. It is conducive to getting out of the dilemma of the fair use system of short video copyright under the current network big data environment.

## 5. Conclusion

Rapid Internet development has created new opportunities for the production, consumption, and dissemination of human creations. Internet users can freely access large information resources in the flawless fair use regime of China's vast cyberspace. The fair use system has been significantly impacted by the development of network technology, which has also resulted in new copyright issues. The existence of the fair use system is founded on the demands of social and economic progress, thus this does not imply that its fundamental principles have changed. It must therefore be continuously developed in accordance with the requirements of modern development if its advantages in preserving the fair use system's equality and its creative zeal are to be fully realised. Therefore, based on the definition of the fair use system of short video copyright, this paper explains the idea of fair use of copyright and the definition and characteristics of short video. It also analyses the challenges and solutions associated with the fair use system of short video copyright in the network environment monitoring and builds a short video repeat detection model using local key points. According to the experimental findings, this algorithm's short video repetition detection accuracy rate can reach 95.8%, and its recall rate can reach 94.5%. Conclusion: Complex scene videos may successfully recognise objects, and they provide a solid data analysis base for the creation of a short video copyright fair use system in the current network context. It is helpful for resolving the fair use system of short video copyright issues in the present big data network environment.

## Figures and Tables

**Figure 1:** Short video UGC, PGC, and PUGC types.

**Figure 2:** System framework.

**Figure 3:** E-R diagram of database.

**Figure 4:** Distribution of downlink average packet size characteristics of seven short video types.

**Figure 5:** Information entropy characteristic distribution diagram of downlink packet size of short video.

**Figure 6:** Speed comparison of various short video repetition detection methods.

**Figure 7:** Recall of various short video repetition detection methods.

**Figure 8:** Accuracy of various short video repetition detection methods.

**Table 1:** Short video service data set.

Short video service type	Number of streams (piece)	Sample bytes (GB)
Tiktok short video	180	6.58
Kwai short video	180	15.24
Microvision	120	34.55
Wechat video number	120	18.69
Youku HD video stream	120	24.85
HTTP video	60	58.75
Kankan video	60	65.58

**Table 2:** Data stream storage format.

Time	Source	Destination	Protocol	Length
0.00000000	117.226.18.29	10.10.143.38	HTTP	1268
0.61587400	Compa1In_d2:57:e2	Broadcast	ARP	60
0.07852500	10.10.142.48	74.125.452.48	SSL	55
0.38568400	10.10.143.38	10.10.143.38	HTTP	1268
0.38564800	118.228.16.29	118.228.16.29	TCP	66
0.38654900	118.228.16.29	10.10.143.38	HTTP	1268
0.38954200	118.228.16.29	10.10.143.38	TCP	54
0.38966800	10.10.143.38	18.228.16.29	TCP	577
0.41254800	118.228.16.29	10.10.143.38	TCP	261

## Data Availability

The data used to support the findings of this study are available from the corresponding author upon request.

## References

[1] Shivakumara P., Wu L., Lu T., Tan C. L., Blumenstein M., Anami B. S. (2017). Fractals based multi-oriented text detection system for recognition in mobile video images. *Pattern Recognition*.

[2] Amanipour V., Ghaemmaghami S. (2019). Median Filtering forensics in compressed video. *IEEE Signal Processing Letters*.

[3] Zheng H., Bai Y., Tian Y. (2022). A multi moving target recognition algorithm based on remote sensing video. *CMES-Computer Modeling in Engineering & Sciences*.

[4] Guang Z., Wang Y., Duan Q. (2022). Evaluation model of urban smart energy system based on improved genetic algorithm-Bp neural network. *International Journal of Pattern Recognition and Artificial Intelligence*.

[5] Yamada H., Yatian T., Nomura H. (2010). Development of network configuration management database system and its application - network management data federation. *Telecommunications System*.

[6] Fang Y., Kang W., Wu Q., Tang L. (2017). A novel video-based over-the-air signature verification system. *Computers and Electrical Engineering*.

[7] Zhang J., Wang K., He Y., Kuang L. (2022). Visual object tracking via cascaded RPN fusion and coordinate attention. *CMES-Computer Modeling in Engineering & Sciences*.

[8] Fund F., Hosseini S. A., Panwar S. S. (2016). Under a cloud of uncertainty: legal questions affecting internet storage and transmission of copyright-protected video content. *IEEE Network*.

[9] Xue L., Wang Y., Wang Q. (2019). Copyright protection of holographic video based on spatiotemporally consistent embedding strategy. *IEEE Transactions on Industrial Informatics*.

[10] Preda R. O., Vizireanu D. N. (2010). A robust digital watermarking scheme for video copyright protection in the wavelet domain. *Measurement*.

[11] Masoumi M., Amiri S. (2013). A blind scene-based watermarking for video copyright protection. *AEU International Journal of Electronics and Communications*.

[12] Lee M. J., Im D. H., Lee H. Y., Kim K. S., Lee H. K. (2012). Real-time video watermarking system on the compressed domain for high-definition video contents: practical issues. *Digital Signal Processing*.

[13] Vizireanu P. D. N. (2011). A robust video watermarking scheme for copyright protection based on human vision system based on wavelet. *Journal of Electronic Imaging*.

[14] Jie J., Yi T., Hua L. (2017). GVoS: A general system for near-repetitive video related applications on storm. *Acm Information System Transactions*.

[15] Wakata S., Shu M. (2015). Brain activity and perception of self-motivation when watching a video of a gripper. *Neural Reports*.

[16] Spelten E. R., Martin L., Gitsels J. T., Pereboom M. T. R., Hutton E. K., van Dulmen S. (2015). Introducing video recording in primary care midwifery for research purposes: procedure, dataset, and use. *Midwifery*.

[17] Chan H. Y., Smidts A., Schoots V. C., Dietvorst R. C., Boksem M. A. S. (2019). Neural similarity at temporal lobe and cerebellum predicts out-of-sample preference and recall for video stimuli. *Neuroimaging*.

[18] Wenwei Z., Yang J. (2010). Video watermarking algorithm based on wavelet transform and neural network. *Programmable Controllers and Factory Automation*.

[19] Zhi S., Zhu Y., Xiao L. (2018). A novel 3D video fingerprinting algorithm based on local feature points. *Chinese Journal of Electronics*.

[20] Lebedev A., Van T. T. (2011). Optimization of high-definition video coding and hybrid fiber-wireless transmission in the 60 GHz band. *Optics Express*.

[21] Erickson N. B., Brenton S. L., Coutts J. N. (2015). Compressed dynamic pattern decomposition for real-time object detection. *Journal of Real-Time Image Processing*.

